# Cyanidin-3-glucoside activates Nrf2-antioxidant response element and protects against glutamate-induced oxidative and endoplasmic reticulum stress in HT22 hippocampal neuronal cells

This article has been retracted.

**DOI:** 10.1186/s12906-020-2819-7

**Published:** 2020-02-11

**Authors:** Monruedee Sukprasansap, Pithi Chanvorachote, Tewin Tencomnao

**Affiliations:** 1 Food Toxicology Unit, Institute of Nutrition, Mahidol University, Salaya campus, 25/25 Phuttamonthon 4 Road, Salaya, Nakhon Pathom, 73170 Thailand; 2 Department of Pharmacology and Physiology, Faculty of Pharmaceutical Sciences, Chulalongkorn University, Bangkok, 10330 Thailand; 3 Cell-based Drug and Health Products Development Research Unit, Faculty of Pharmaceutical Sciences, Chulalongkorn University, Bangkok, 10330 Thailand; 4 Age-Related Inflammation and Degeneration Research Unit, Department of Clinical Chemistry, Faculty of Allied Health Sciences, Chulalongkorn University, Bangkok, 10330 Thailand

**Keywords:** Cyanidin-3-glucoside, Anthocyanin, Oxidative stress, ER stress, Glutamate, Nrf2, Antioxidant enzyme, Neuroprotective effect, HT22 cells

## Abstract

**Background:**

Cyanidin-3-glucoside (C3G), a major anthocyanin present in berries, exhibits a strong antioxidant and has been shown to possess a neuroprotection. Prolonged exposure to glutamate will lead to oxidative damage and endoplasmic reticulum stress which could play a key detrimental role in the development of neurodegenerative disorders (NDs). In the present study, we investigated the neuroprotective effect and underlying mechanisms of C3G on the reduction of oxidative/ER stress-induced apoptosis by glutamate in HT22 mouse hippocampal neuronal cells.

**Method:**

Cells were pre-treated with C3G in various concentrations, followed by glutamate. Cell viability and toxicity were examined using MTT and LDH assays. The apoptotic and necrotic cell death were carried out by Annexin V-FITC/propidium iodide co-staining assays. Generation of intracellular reactive oxygen species (ROS) in cells was measured by flow cytometry using DCFH-DA probe. Expression of antioxidant genes was evaluated by Real-time polymerase chain reaction analysis. The possible signaling pathways and proteins involved were subsequently demonstrated by Western blot analysis.

**Result:**

The pretreatment of the HT22 cells with C3G protected cell death from oxidative toxicity induced by glutamate. We demonstrated that treatment cells with glutamate caused several radical forms of ROS formation, and they were abolished by specific ROS inhibitors. Interestingly, C3G directly scavenged radical activity and inhibited intracellular ROS generation in our cell-based system. In addition, C3G pretreatment suppressed the up-regulation of specific ER proteins namely calpain, caspase-12 and C/EBP homologous proteins (CHOP) induced by glutamate-mediated oxidative and ER stress signal by up-regulating the expressions of survival proteins, including extracellular regulated protein kinase (ERK) and nuclear factor E2-related factor 2 (Nrf2). Furthermore, dramatically activated gene expression of endogenous antioxidant enzymes (i.e. superoxide dismutases (SODs), catalase (CAT) and glutathione peroxidase (GPx)), and phase II enzymes (glutathione-S-transferases (GSTs)) was found in C3G-treated with cells.

**Conclusions:**

Our finding suggest that C3G could be a promising neuroprotectant via inhibition of glutamate-induced oxidative and ER stress signal and activation of ERK/Nrf2 antioxidant mechanism pathways.

## Background

The growing incidence and prevalence of the neurodegeneration are still in the absence of effective therapeutic interventions and obscure understanding of mechanism and pathophysiology of the disease states. Neurodegenerative disorders (NDs) are characterized by dysfunction, damage and death of neurons, resulting in the progressive deterioration of the structure and cognitive functions in brain. This process pathway is obviously found in the brain aging. The damage observed in aging is exacerbated in NDs such as dementia and Alzheimer’s diseases (AD) [1, 2]. Oxidative stress is also known as a central mechanism in the pathogenesis of AD. Therefore, oxidative stress-mediated neuronal death has received much attention in the search for underlying mechanisms and potential therapeutic targets. Several lines of evidence found that oxidative stress increases in the brain during aging process. The hypothesis of oxidative stress assumes that a disruption in the balance of reactive oxygen species (ROS) causes an oxidative damage of the cellular macromolecules including the oxidations and modifications of DNA and protein, and the induction of lipid peroxidation, thus ultimately resulting in cell death in nervous system [3–5]. Although it is the main excitatory neurotransmitter in neurons, excessive accumulation of glutamate can not only activate ROS production and oxidative neurotoxicity contributing to neuronal apoptosis [1, 6], but associate with acute and chronic NDs as well [7, 8]. Multiple lines of evidence have supported that glutamate-induced apoptosis relates to the cysteine uptake through the cysteine/glutamate antiporter channel, leading to the diminution of endogenous antioxidant glutathione and increase of ROS in neurons [9–11].

The approach of oxidative-endoplasmic reticulum (ER) stress mechanism has considered the most crucial signal causing NDs [8, 11–14]. ER stress plays a pivotal part in the progression of NDs [15–18]. Mechanisms involving in signaling of ER stress-induced apoptosis have been suggested to associate with the calpain activation. It is a calcium-dependent neutral protease, leading to the initiation of caspase-12 proteolytic activity [19–21]. Calpain and caspase-12 have been known as specific ER stress markers and unfolded protein response (UPR) [15–17, 19–21]. Besides, CHOP (C/EBP-homologous protein, GADD153) has been reported to upregulate the protein expression in the cells undergoing ER stress [12, 16, 22]. This elongation process and activation of CHOP have been shown to not only inhibit the anti-apoptotic BCL2 family proteins expressed, but also stimulate the transcription of pro-apoptotic BCL2 family members expression leading to apoptosis, which functions as an integrator and amplifier of the mechanistic approach of cell death [11–13, 22–24].

Numerous reports using experimental models of different disorders suggest that nuclear factor E2-related factor2 (Nrf2) pathway activation represents a promising therapeutic approach to restore the systemic and neuronal redox balance by reducing ROS-mediated neuronal damage [25]. It has been reported that Nrf2 signaling promotes a survival in response to ER stress in neurons [16, 18]. Nrf2 has the function as a key endogenous antioxidants and phase II detoxification enzymes systems for increasing cellular defense against oxidative stress [26, 27]. However, only a few Nrf2-activating compounds have been tested in a clinical setting. Additionally, it has been demonstrated that Nrf2 is activated by the mitogen-activated protein kinases (MAPKs) signaling under conditions of oxidative stress [8, 28, 29]. With respect to the MAPKs signaling such as extracellular-regulated kinases (ERKs), has been originally shown to be involved in the stress response and important for cell survival because of anti-apoptotic signals in neuronal cells [13, 30–32].

Recognized as a natural phyochemical in the family of the anthocyanins, Cyanidin-3-glucoside (C3G) produces the red, purple and blue pigments seen in many edible plants, particularly rich in berry fruits. C3G has been reported to benefit health through a vast range of biological effects including antioxidant, anti-inflammatory, anti-ischemic, and anti-cancer properties [25, 33–37]. C3G and other anthocyanins were observed in the cerebellum, cortex, hippocampus or striatum of the blueberry supplementation rats, but not the controls [38]. Importantly, C3G can also cross the blood brain barrier and localize in numerous brain regions critical for learning and memory, which are neuroavailable, as well, with anthocyanins residing in tissue longer than in plasma [38–40]. Several lines of evidence have demonstrated that C3G not only blocked ethanol-mediated intracellular accumulation of ROS, but also inhibited ER stress-induced neuronal cell death and it reversed ethanol-induced inhibition of neurite outgrowth [41, 42]. Anthocyanin in the form of C3G was shown to upregulate glutamate-cysteine ligase expression, which in turn mediated the decrease in ROS levels [43]. C3G protected human umbilical vein endothelial cells from oxidative stress by triggering Nrf2 and activating the cellular antioxidant pathway [44]. Neuroprotective mechanism of C3G against glutamate-induced neuronal cells apoptosis through ER stress has never been well understood. Here, we investigate the effect and underlying mechanism by which C3G protect against glutamate-mediated neurotoxicity via oxidative-ER stress pathway and examined the function of endogenous antioxidant system through ERK/Nrf2 signaling pathway.

## Methods

### Chemicals and reagents

C3G (purity ≥99%, Fig. 1), L-glutamic acid, Dulbecco’s modified Eagle medium (DMEM), 2, 2-diphenyl-1-picrylhydrazyl (DPPH) and fetal bovine serum (FBS) were purchased from Sigma-Aldrich Co. (St Louis, MO, USA). Antibodies against calpain, caspase12, CHOP, ERK, p-ERK (Thr202/Tyr204), β-actin and horseradish peroxidase-coupled secondary antibodies were purchased from Cell Signaling Technology (Danvers, MA, USA), and Nrf2 was obtained from Santa Cruz Biotechnology (Dallas, TX, USA). 3-(4,5-dimethylthiazol-2-yl)-2, 5-diphenyltetrazolium bromide (MTT) was purchased from Bio basic (Toronto, Canada). Dimethylsulfoxide (DMSO) was purchased from Merck (Darmstadt, Germany). Penicillin-streptomycin solution was obtained from Corning Inc. (Corning, NY, USA). Annexin V FITC/PI kit was purchased from Biolegend (San Diego, CA, USA). The reagent kit for lactate dehydrogenase (LDH) was bought from Promega’s CytoTox 96™ (Madison, WI, USA) and 2′,7′- dichlorofluorescein diacetate (H_2_DCF-DA) was obtained from Life technology (Carlsbad, CA, USA). Trizol was purchased from Invitrogen (Carlsbad, CA, USA).

**Fig. 1:** Chemical structure of C3G

### Preparation of C3G solution

To prepare the stock solution of 100 mM, C3G was dissolved in DMSO. Dilutions of C3G were made in DMEM according to the concentrations required. The cells were pre-incubated with C3G for 24 h before addition of glutamate.

### Cell culture

Mouse hippocampal neuronal (HT22) cell line was kindly provided by Prof. David Schubert (The Salk Institute, San Diego, CA, USA). HT22 cells were cultivated in DMEM at 37 °C in a 5% CO_2_ humidified incubator. The medium for culture containing 10% FBS and 100 U/ml penicillin/streptomycin was used.

### MTT assay

Cell viability was determined using a colorimetric MTT assay. Five thousand cells in 100 μl of DMEM medium were seeded onto each well of 96-well plates and incubated overnight. Next, the cells were treated with various doses of C3G (0–100 μM) for 24 h. The treated cells were incubated with 500 μg/ml of MTT at 37 °C for 4 h. After the supernatant was removed, formazan product was solubilized in DMSO. The MTT product was read using a microplate reader at 550 nm. The percentage of cell viability was calculated and compared with non-treated control cells.

### LDH assay

The cellular cytotoxicity of cell death was measured using CytoTox 96™ assay kit following the manufacturer’s protocol. In order to detect LDH released from damaged cells, we followed the instruction described previously [14]. After the specified treatment and time, the culture supernatant was incubated with substrate mix for 30 min in the dark at room temperature, and then the stop solution was added. The absorbance at 490 nm was measured using a microplate reader. Data were expressed as percentage of maximum LDH release activity of cells.

### Apoptosis assay

Cells were evaluated by the fluorescein isothiocyanate (FITC)-annexin V apoptosis detection kit with PI to quantify apoptotic and necrotic cell death, respectively, according to the manufacturer’s protocol. The treatment cells were incubated with Annexin V-FITC reagent and then PI solution for 15 min at room temperature in the dark. Subsequently, the binding buffer was added to mark the final volumes. The cells were analyzed using flow cytometry (FACSCalibur, BD Biosciences, San Jose, CA, USA).

### Intracellular ROS assay

An intracellular ROS production was determined by DCFH_2_-DA probe. In brief, the cells were pre-treated with various concentrations of C3G for 24 h, followed by glutamate for 18 h. Subsequently, the treated cells were incubated with 10 μM DCFH_2_-DA for 45 min at 37 °C. After the completed condition, the cells were washed, trypsinized and resuspended in buffer. The fluorescence intensity was detected by flow cytometry (FACSCalibur, BD Biosciences, San Jose, CA, USA) using excitation and emission wavelengths of 488 nm and 525 nm, respectively.

### Free radical 2, 2-diphenyl-1-picrylhydrazyl (DPPH) scavenging assay

The procedure of free radical scavenging method was measured as described previously [45]. The C3G were added in a 96-well plate, followed by 150 μM DPPH reagent in 80% methanol. The plate was performed in the dark at room temperature for 30 min. After that, the plate was read at 520 nm using microplate reader. As a standard antioxidant, Trolox solution was used. Data were expressed as the percentage of scavenging activity. It was calculated according to the following formula: % Radical Scavenging activity = [100 × (A - B) -C]/C, where: A = sample absorbance 520 nm; B = blank absorbance 520 nm; C = control absorbance 520 nm.

### Western blot analysis

The protein expression was determined by Western blotting. Briefly, HT22 cells were seeded onto 6-well plate at density of 2 × 10^5^ cells/well for overnight, and were treated with different doses of C3G or glutamate. After the treatment, the cells were washed twice with ice-cold phosphate buffered saline. Next, the specific treatment cells were performed in lysis buffer containing 20 mM Tris·HCl (pH 7.5), 1% Triton X, 150 mM sodium chloride, 10% glycerol, 1 mM sodium orthovanadade, 50 mM sodium fluoride, 100 mM phenylmethylsulfonyl fluoride and commercial protease inhibitor cocktail (Roche Diagnostics GmbH, Mannheim, Germany) for 45 min on ice. The cell lysates were collected by scraping from each well-plate, and then the mixture was centrifuged at 12,000 x g for 20 min. This supernatant was measured the protein concentration using the Bradford protein assay (Bio-Rad laboratories, Hercules, CA, USA). Equal amount of protein samples (40 μg) were denatured by heating in Laemmli loading buffer at 95 °C for 5 min and subsequently loaded onto a 10% SDS-PAGE and transferred to PVDF membranes (Bio-Rad Laboratories). Transferred membranes were blocked for 1 h in 5% nonfat dry milk in TBST (25 mM Tris-HCl, pH 7.5, 125 mM NaCl, and 0.05% Tween 20) and incubated with specific primary antibodies against calpain 1 Large (diluted 1:1000), caspase12 (diluted 1:1000), CHOP (D46F1) (diluted 1:1000), ERK (137F5) (diluted 1:25000), p-ERK (Thr202/Tyr204) (D13.14.4E) (diluted 1:16000), Nrf2 (C-20): sc-722 (diluted 1:8000) or β-actin (13E5) (diluted 1:16000) at 4 °C overnight. Membranes were washed with TBST for 15 min and incubated with horseradish peroxidase-coupled secondary antibodies (diluted 1:16000) for 1 h at room temperature. Next, the specific protein bands were visualized using a film exposure with the chemiluminescence detection system (ECL™ Select Western blotting detection reagent: GE Healthcare, Piscataway, NJ, USA) and quantified using Image J software.

### RNA isolation and real-time PCR analysis

This method was performed as described previously [14]. In brief, total RNA was isolated from specific treatment cells using Trizol reagent (Invitrogen, Carlsbad, CA, USA). cDNA was synthesized from 1 μg of total RNA using Accupower RT Premix (Bioneer, Daejeon, Korea) with oligo-dT primers following the manufacturer’s instructions. Each real-time PCR reaction was performed using the Exicycler Real Time Quantitative Thermal Block (Bioneer) and SYBR Green was used for the detection of double-stranded DNA. Quantitative real-time PCR experiments for specific genes were carried out using Green Star PCR Master Mix (Bioneer). The specific sequence of primers were SOD1 forward (5′-CAGGACCTCATTTTAATCCTCAC-3′) SOD1 reverse (5′-CCCAGGTCTCCAACATGC-3′), SOD2 forward (5′-CTGGACAAACCTGAGCCCTA-3′) SOD2 reverse (5′-TGATAGCCTCCAGCAACTCTC-3′), CAT forward (5′-CAGCGACCAGATGAAGCA-3′) CAT reverse (5′-CTCCGGTGGTCAGGACAT-3′), GPx forward (5′-ACAGTCCACCGTGTATGCCTTC-3′) GPx reverse (5′-CTCTTCATTCTTGCCATTCTCCTG-3′), GSTo1 forward (5′-CAGCGATGTCGGGAGAAT-3′) GSTo1 reverse (5′-GGCAGAACCTCATGCTGTAGA-3′), GSTa2 forward (5′-TCTGACCCCTTTCCCTCTG-3′) GSTa2 reverse (5′-GCTGCCAGGATGTAGGAACT-3′) and β-actin forward (5′-GGCTGTATTCCCCTCCATCG-3′) β-actin reverse (5′-CCAGTTGGTAACAATGCCATGT-3′) [46]. All gene transcripts were measured and fluorescent signals were measured in real time-PCR experiments under the following conditions: the initial denaturation step at 95 °C for 15 min, followed by 45 cycles at 95 °C for 15 s and primer annealing/extension at 55 °C for 30 s. Melting curve analysis was performed to verify primer specificity. The relative expression of each gene was normalized to the internal control gene (β-actin).

### Statistical analysis

Data are mean ± S.D. from at least three independent experiments. Statistical analysis was performed by one-way analysis of variance ANOVA followed by Dunnett’s post hoc test at a significant level of *p* < 0.05 using SPSS version 22.

## Results

### C3G inhibits glutamate-induced cytotoxicity in mouse hippocampal neuronal cells

Treatment of the cells with C3G in various concentrations (0–100 μM) for 24 h did not cause obvious cytotoxicity compared with the non-treated control cells. These results indicated that C3G was relatively non-cytotoxic at the tested concentration in our HT22 cell model (Fig. 2a). Next, pretreated cells with 0–100 μM C3G for 24 h, followed by 5 mM glutamate for 18 h, and cell viability was assessed using MTT assay. Treatment of the cells with C3G (0.05–1 μM) attenuated the glutamate-induced toxicity in a dose-dependent manner with the highest protective effect at 1 μM (Fig. 2b). Furthermore, the results were confirmed by cell death LDH assay (Fig. 2c). We found that glutamate caused injured cells and the pretreatment cells with C3G (0.05–1 μM) significantly inhibited such cell deaths. Thus, C3G concentrations ranging from 0.05 to 1 μM were chosen for subsequent experiments with regard to cell treatment.

**Fig. 2:** Protective effect of C3G against glutamate-mediated cytotoxicity and cell death in HT22 cells. (**a**) Cells were treated with C3G (0–100 μM) for 24 h. Cell viability was evaluated by MTT assay. (**b**) After indicated treatment for 24 h, followed by 5 mM glutamate for 18 h, cell viability was detected using the MTT assay and (**c**) cell death was measured using LDH assay. (**d**) Cells were pretreated C3G (0–1 μM) and followed by 5 mM glutamate, mode of cell death was examined by Annexin V-FITC/PI double staining, and analyzed using flow cytometry. The cell population at different stages are shown. (**e**) Histogram represents the percentage of cell death (white bar: apoptosis and black bar: necrosis). (**f**) Morphology of treated cells were observed under microscope (scale bar is 50 μm). The data are expressed as mean ± SD (*n* = 4). ^#^*p* < 0.05 versus non-treated control, ^*^p < 0.05, ^**^p < 0.01, ^***^p < 0.001 versus 5 mM glutamate-treated cells

Additionally, to further verify the mode of cell death from cytotoxic results above, apoptosis and necrosis were judged by Annexin V-FITC and propidium iodide co-staining approach. Cells were pretreated with various concentrations of C3G with (0.05–1 μM) for 24 h, followed by 5 mM glutamate for 18 h. The cell apoptosis and necrosis were quantified using flow cytometry. Our result showed that cells treated with glutamate resulted in the approximately 45 and 3% of apoptotic and necrotic cell death, respectively. We found that C3G clearly protected against glutamate-induced apoptosis with the maximum protective effect could be distinguished at the concentration of 1 μg/ml (Fig. 2d and e). In addition, cell morphology was observed under a phase contrast microscopy (Fig. 2f). The glutamate-treated cells showed round, shrink and lost elongated neuron shapes, while pretreatment the cells with C3G improved the native morphology as observed in the non-treated control. These results suggest that C3G exerts the neuroprotective effect against glutamate-induced cell death in HT22 hippocampal neuronal cells.

### C3G suppresses the intracellular ROS production by glutamate and its antioxidant activity

Glutamate has been well recognized to induce neuronal cell death via oxidative stress-dependent mechanism. To elucidate the effect of C3G on glutamate-induced oxidative stress, the intracellular ROS level in HT22 cells was determined using DCFH_2_-DA probe. HT22 cells were pretreated with different concentrations of C3G for 24 h and then exposed to glutamate for 18 h. The fluorescence intensity was measured by flow cytometry. We found that pretreatment of the cells with C3G significantly diminished the levels of ROS induced by glutamate as shown in Fig. 3a and b, while the glutamate treatment alone led to dramatic increase in cellular ROS level compared to the non-treated control cells. Additionally, we demonstrated the antioxidant activity of C3G using DPPH radical scavenging assay. The result showed that C3G had relatively potent ability to scavenge the radical in a dose-dependent fashion (Fig. 3c). Furthermore, the ROS-inducing effect of glutamate-induced oxidative toxicity could be inhibited by specific ROS inhibitors namely, 5 mM N-acetyl-L-cysteine (NAC); total radical inhibitor, 5 mM glutathione (GSH) and 7500 Unit/mg catalase (CAT); hydrogen peroxide inhibitors, 50 μM Mn (III) tetrakis (4-benzoic acid) porphyrin (MnTBAP); superoxide anion inhibitor, and 1 mM deferoxamine mesylate (DM); hydroxyl radical inhibitor. Each inhibitor was pretreated with cells prior to addition with 5 mM glutamate, and MTT assay was performed. Our data displayed that treatment cells with the glutamate caused the all of radical species upregulated in the HT22 cells and such event could be abolished by the addition of these specific inhibitors, confirming that the all of ROS formation species can be induced by glutamate treatment in our system (Fig. 3d). These results indicate that C3G inhibits glutamate-induced ROS generation and also directly scavenges the reactive oxygen radicals.

**Fig. 3:** Effect of C3G on glutamate-induced ROS generation in HT22 cells and antioxidant activity. (**a**) The pretreatment of cells with C3G (0-1 μM) for 24 h, followed by 5 mM glutamate for 18 h. After that the cells were incubated with 10 μM DCFH_2_-DA for 45 min at 37 °C. The fluorescence intensity was measured by flow cytometry. (**b**) Data were expressed as a relative ROS level of non-treated control. (**c**) The free radical scavenging activity of various concentrations of C3G (0.05–1 μM) was evaluated using DPPH assay. (**d**) Cells were pretreated specific ROS inhibitors for 30 min and followed by 5 mM glutamate for 18 h, cell viability was detected by the MTT assay. Glu, glutamate; NAC, N-acetyl-L-cysteine; GSH, glutathione; CAT, catalase; MnTRAP, Mn (III) tetrakis (4-benzoic acid) porphyrin; DM, deferoxamine mesylate. Values are the mean ± SD (n = 4). ^#^p < 0.05 versus non-treated control, ^*^p < 0.05, ^**^p < 0.01, ^***^p < 0.001 versus 5 mM glutamate-treated cells

### C3G attenuates the specific-ER stress apoptosis signaling in glutamate-induced neuronal cell death

To further illustrate the effect of C3G on glutamate-induced neuronal cell death mediated through oxidative and ER stress, the protein expression of specific-ER stress markers including the calcium ion-mediated calpain, caspase-12 and CHOP was perforumed using Western blot analysis. Cells were pre-treated with various concentrations of C3G (0.05–1 μM) for 24 h and followed by glutamate for 18 h. Figure 4 reveals that the treated cells with glutamate alone significantly increased the protein expression of not only calpain, but also cleaved caspases-12 and CHOP. Moreover, C3G pretreatment significantly reduced the expression of all apoptotic ER stress proteins namely calpain, cleaved caspase-12 and CHOP (Fig. 4). These results suggest that C3G has an ability to suppress glutamate-induced oxidative/ER stress apoptosis signaling in HT22 cells.

**Fig. 4:** Protective effect of C3G against glutamate-induced ER stress apoptotic protein expression in HT22 cells. Cells were pretreated with C3G (0–1 μM) for 24 h, followed by 5 mM glutamate for 18 h. After treatment, (**a**) the level of calpain, caspase-12 and CHOP were determined by Western blot analysis, and β-actin was served as the loading control. (**b**, **c**, **d**) Relative protein levels were quantified by densitometry and the mean data from independent experiments were normalized to the results. The data represent the means of four independent samples ± SD. ^#^*p* < 0.05 versus non-treated control, ^*^p < 0.05, ^**^p < 0.01, ^***^p < 0.001 versus 5 mM glutamate-treated cells

### C3G up-regulates ERK and Nrf2 antioxidant signaling proteins

Nrf2 is known to play an essential role in endogenous antioxidants and phase II detoxification enzymes systems for increasing cellular defense against oxidative stress [26, 27]. Nrf2 pathway activation represents a promising therapeutic approach to restore the systemic and neuronal redox balance by reducing ROS-mediated neuronal damage [25]. In addition, it has been demonstrated that Nrf2 is activated by the MAPKs signaling under conditions of oxidative stress, namely ERK which has been originally shown that are also involved in the stress response and an important for cell survival in role of anti-apoptotic signals in neuronal cells [13, 28–32, 47]. Therefore, we investigate the protective effect of C3G on oxidative/ER stress-mediated cell death in the HT22 cell model. The expression of ERK and Nrf2 proteins in response to the cell treatment was assessed by Western blot analysis. The cells were treated with various concentrations of C3G (0.05–1 μM) for 24 h. We found that C3G treatment led to a significant increase in Nrf2 protein level, while the p-ERK/ERK protein level was found to be slightly increased (Fig. 5). Our results suggest that C3G activates the ERK/Nrf2 targeted-antioxidant protein signaling.

**Fig. 5:** Effect of C3G on ERK and Nrf2 antioxidant regulatory proteins in HT22 cells. Cells were pretreated with C3G (0–1 μM) for 24 h, followed by 5 mM glutamate for 18 h. After treatment, (**a**) the expression levels of p-ERK, ERK and Nrf2 were determined by Western blot analysis, and β-actin was served as the loading control. (**b**) Relative protein levels were quantified by densitometry and the mean data from independent experiments were normalized to the results. The data represent the means of four independent samples ± SD. ^#^*p* < 0.05 versus non-treated control, ^*^p < 0.05, ^**^p < 0.01, ^***^p < 0.001 versus 5 mM glutamate-treated cells

### C3G up-regulates antioxidant enzymes and phase II detoxifying enzymes gene expressions

To further confirm the antioxidant mechanism of action of C3G against glutamate-induced ROS and apoptosis in our HT22 cell model, we determined the gene expressions of antioxidant enzymes (SODs, CAT, and GPx) and phase II enzymes (GSTs) using real-time PCR analysis. Cells were treated with various concentrations of C3G (0.05–1 μM) for 24 h. Our results showed that C3G treatment significantly increased the gene expressions of antioxidant enzymes including SODs (SOD1 and SOD2), CAT and GPx, as well as the gene expressions of phase II enzyme, namely GSTs (GSTo1 and GSTa2) in a dose-dependent manner (Fig. 6). Taken together, these finding indicate that the C3G can up-regulate the cellular antioxidant and phase II detoxifying enzymes which they act as a downstream mechanism targets of Nrf2, providing as a possible neuroprotective mechanism of C3G against oxidative toxicity.

**Fig. 6:** Effect of C3G on the gene expression of endogenous antioxidant and phase II enzymes in HT22 cells. After treatment cells with C3G (0–1 μM), cells were collected and analyzed for gene expression. The levels of (**a**) SOD1, (**b**) SOD2, (**c**) CAT, (**d**) GPx, (**e**) GSTo1 and (**f**) GSTa2 mRNA expression were determined by quantitative real-time PCR. The data are shown as fold change of mRNA expression normalized with β-actin. Values are mean ± SD (n = 4). ^#^p < 0.05 versus non-treated control, ^*^p < 0.05, ^**^p < 0.01, ^***^p < 0.001 versus 5 mM glutamate-treated cells

## Discussion

One of the most significant pathologies involving neuronal cell death in neurodegeneration is oxidative stress which may occur under the influence of inflammation and cellular stress in neurons. Various lines of evidence have suggested that the production and accumulation of ROS and ER stress death signaling pathway have been shown to play a crucial mechanism in triggering neuronal death [13, 16–18, 48]. Although glutamate, the neurotransmitter in the mammalian central nervous system, plays a major role in many brain functions, it can cause neurotoxicity at prolonged or high concentration resulting in oxidative stress-mediated cell death in neurons. This impact leads to various neurodegenerative diseases such as AD. Several previous reports revealed that glutamate-induce ROS production and ROS-based ER stress apoptosis signaling are major factors in the progression of HT22 cell death [8, 11, 49]. Neuronal cells are particularly susceptible to oxidative stress, resulting in damaged cell and death, as these cells possess low levels of endogenous antioxidant system [6]. Also, the antioxidants and natural compounds that have a potent action in inhibition of ROS production, ROS detoxification, or direct interact with the ROS produced by glutamate are probably to defend against glutamate-mediated neuronal cell death. Therefore, glutamate-induced oxidative and ER stress can also cause cell apoptosis in neurons [12, 14, 38, 42].

As expected, the present study clearly showed that glutamate treatment could generate the intracellular ROS and ER stress resulting in cell apoptosis in our HT22 mouse hippocampal cell model. Consequently, we examined the protein expressions of apoptotic-ER stress markers including calpain, caspase-12 and CHOP in response to glutamate treatment, confirming that glutamate-induced oxidative stress is an essential mechanism linking ER stress to apoptosis in these cells. For neuroprotective effect, the results revealed that treatment of cells with non-toxic concentrations of C3G protected against glutamate-induced cell apoptosis. In the current study, we found that HT22 cells facing glutamate showed higher levels of ROS and C3G inhibited the generation of ROS. Remarkably, the addition of C3G could be able to suppress all ER stress proteins in glutamate-treated cells. This neuroprotective effect involved in a powerful antioxidant property of the C3G, oxidative stress is well known as a main inducer of ER stress by influencing intracellular calcium ions release from ER, contributing to calpain and caspase-12 activations [19, 20]. The caspase-12 is a specific caspase of ER stress signal that it is activated by the function of calpain [13, 18, 21, 50]. Furthermore, we investigated the activation of another ER stress marker namely CHOP, regulating protein in glutamate-treated HT22 cells. Physiologically, the CHOP is stored at a low level, but it is up-regulated in the nucleus under ER stress condition [14, 15, 17, 24]. We have discovered that C3G could decrease all of ER stress markers induced by glutamate, assuring that this C3G-anthocyanin type exerts a potent neuroprotection by reduction of ER stress signal molecules.

Collectively, these findings showed that C3G acted as a neuroprotector in mouse hippocampal HT22 cells experimental model. Our results suggested that C3G can significantly decrease glutamate-induced oxidative/ER stress, resulting in apoptosis, by blocking the intracellular ROS generation and enhancing the antioxidant system. Further, we investigated that the protective effect of C3G that not only exerted its antioxidant activity through the direct scavenging property, which inhibited intracellular ROS generation, but C3G also enhanced the expression of Nrf2 antioxidant protein by MAPK/ERK signaling. Besides, we found that pretreatment of the cells with C3G markedly up-regulated the expression of antioxidant enzymes, namely SOD, CAT, GPx and GST which are the downstream function of Nrf2 [26, 27, 47] and these antioxidant enzymes found in brain tissue for ROS detoxification [2–4, 25–27, 31, 51]. C3G, this anthocyanin has recently gained attention for its multifunctional benefits including antioxidant property, anti-inflammation and prevention of neurodegenerative disorders [27, 51–53]. It is also able to reach the brain, which probably to penetrate the blood brain barrier as they can be found in various part of the brain such as hippocampus, cerebellum, cortex, or striatum of the rats after berry feeding [38, 54–57]. Interestingly, it has revealed that C3G up-regulated glutamate-cysteine ligase expression, resulting in the decrease of intracellular ROS levels [43]. Recently, some work has focused on C3G blocked oxidative stress by inducing Nrf2 and enhancing the cellular antioxidant pathway in human umbilical vein endothelial cells [44]. Previous studies have demonstrated that activation of the Nrf2 pathway protect neurons against oxidative stress from glutamate- and H_2_O_2_-induced cell death [58, 59]. Supporting evidence has found that dimethyl fumarate protected neural stem/progenitor cells and neurons from H_2_O_2_-induced oxidative damage through Nrf2-ERK1/2 MAPK pathway [60].

## Conclusion

The present study demonstrated that C3G inhibited glutamate-induced oxidative/ER stress mediated HT22 neuronal cell apoptosis by suppressing ROS, up-regulating antioxidant and phase II enzymes system via enhancing the ERK/Nrf2 signaling pathway. Our research findings support the potential benefit of C3G for the prevention of neurodegenerative diseases. The current findings for the protective mechanism of C3G in HT22 neuronal cell model is summarized in Fig. 7. Therefore, C3G is a promising candidate for further investigation as a neuroprotective strategy.

**Fig. 7:** Summary diagram of the proposed mechanisms underlying protective effects of C3G against glutamate-induced oxidative/ER stress apoptosis in HT22 cells. Prolonged glutamate-induced ROS production stimulates oxidative stress lead to ER stress. The resultant oxidative stress activate the specific ER stress apoptosis mechanisms involving calcium ion-mediated calpain activation contribute to caspase-12 cascades apoptosis signal, together with CHOP apoptosis pathway. C3G is able to reduce ROS and trigger survival marker proteins including p-ERK/ERK and Nrf2 expression, leading to an increase level of the endogenous antioxidant and phase II detoxifying enzymes function. As a consequence, these effects resulted in the inhibition of apoptotic-ER stress signaling proteins and enhancing HT22 neuronal cell survival via the ERK/Nrf2 signaling pathway

## Data Availability

All data are analyzed and contained within the manuscript. The datasets used and/or analyzed during the current study are available from the corresponding author on reasonable request.

## Abbreviations

AD: Alzheimer’s disease
C3G: cyanidin-3-glucoside
CAT: catalase
CHOP: C/EBP homologous proteins
DCFH2-DA: 2′,7′- dichlorofluorescein diacetate
DPPH: 2, 2-diphenyl-1-picrylhydrazyl
ER: endoplasmic reticulum
Glu: glutamate
GPx: glutathione peroxidase
GST: glutathione-S-transferase
LDH: Lactate dehydrogenase
MTT: 3-(4,5-dimethylthiazol-2-yl)-2,5-diphenyltetrazolium bromide
Nrf2: nuclear factor E2-related factor2;
PI: propidium iodide
ROS: reactive oxygen species
SOD: superoxide dismutase
UPR: unfolded protein response

## References

[1] Zhu X, Raina AK, Lee HG, Casadesus G, Smith MA, Perry G (2004). Oxidative stress signalling in Alzheimer's disease. Brain Res.

[2] Markesbery William R., Carney John M. (2006). Oxidative Alterations in Alzheimer's Disease. Brain Pathology.

[3] Butterfield DA, Perluigi M, Sultana R (2006). Oxidative stress in Alzheimer's disease brain: new insights from redox proteomics. Eur J Pharmacol.

[4] Maher P, Schubert D (2000). Signaling by reactive oxygen species in the nervous system. Cellular and molecular life sciences : CMLS.

[5] Pratico D (2008). Oxidative stress hypothesis in Alzheimer's disease: a reappraisal. Trends Pharmacol Sci.

[6] Jia J, Xiao Y, Wang W, Qing L, Xu Y, Song H, Zhen X, Ao G, Alkayed NJ, Cheng J (2013). Differential mechanisms underlying neuroprotection of hydrogen sulfide donors against oxidative stress. Neurochem Int.

[7] Greenwood SM, Connolly CN (2007). Dendritic and mitochondrial changes during glutamate excitotoxicity. Neuropharmacology.

[8] Jin ML, Park SY, Kim YH, Oh JI, Lee SJ, Park G (2014). The neuroprotective effects of cordycepin inhibit glutamate-induced oxidative and ER stress-associated apoptosis in hippocampal HT22 cells. Neurotoxicology.

[9] Ha JS, Park SS (2006). Glutamate-induced oxidative stress, but not cell death, is largely dependent upon extracellular calcium in mouse neuronal HT22 cells. Neurosci Lett.

[10] Jeong GS, Byun E, Li B, Lee DS, Kim YC, An RB (2010). Neuroprotective effects of constituents of the root bark of Dictamnus dasycarpus in mouse hippocampal cells. Arch Pharm Res.

[11] Yang EJ, Lee JY, Park SH, Lee T, Song KS (2013). Neuroprotective effects of neolignans isolated from Magnoliae cortex against glutamate-induced apoptotic stimuli in HT22 cells. Food and chemical toxicology : an international journal published for the British Industrial Biological Research Association.

[12] Choi JH, Choi AY, Yoon H, Choe W, Yoon KS, Ha J, Yeo EJ, Kang I (2010). Baicalein protects HT22 murine hippocampal neuronal cells against endoplasmic reticulum stress-induced apoptosis through inhibition of reactive oxygen species production and CHOP induction. Exp Mol Med.

[13] Doyle KM, Kennedy D, Gorman AM, Gupta S, Healy SJ, Samali A (2011). Unfolded proteins and endoplasmic reticulum stress in neurodegenerative disorders. J Cell Mol Med.

[14] Sukprasansap M, Chanvorachote P, Tencomnao T (2017). Cleistocalyx nervosum var. paniala berry fruit protects neurotoxicity against endoplasmic reticulum stress-induced apoptosis. Food Chem Toxicol.

[15] Bernales S, Soto MM, McCullagh E (2012). Unfolded protein stress in the endoplasmic reticulum and mitochondria: a role in neurodegeneration. Front Aging Neurosci.

[16] Chaudhari N, Talwar P, Parimisetty A, Lefebvre d'Hellencourt C, Ravanan P (2014). A molecular web: endoplasmic reticulum stress, inflammation, and oxidative stress. Front Cell Neurosci.

[17] Lee JH, Won SM, Suh J, Son SJ, Moon GJ, Park UJ, Gwag BJ (2010). Induction of the unfolded protein response and cell death pathway in Alzheimer's disease, but not in aged Tg2576 mice. Exp Mol Med.

[18] Liu D, Zhang M, Yin H (2013). Signaling pathways involved in endoplasmic reticulum stress-induced neuronal apoptosis. The International journal of neuroscience.

[19] Lamkanfi M, Kalai M, Vandenabeele P (2004). Caspase-12: an overview. Cell Death Differ.

[20] Momoi T (2004). Caspases involved in ER stress-mediated cell death. J Chem Neuroanat.

[21] Nakagawa T, Zhu H, Morishima N, Li E, Xu J, Yankner BA, Yuan J (2000). Caspase-12 mediates endoplasmic-reticulum-specific apoptosis and cytotoxicity by amyloid-beta. Nature.

[22] Ghosh AP, Klocke BJ, Ballestas ME, Roth KA (2012). CHOP potentially co-operates with FOXO3a in neuronal cells to regulate PUMA and BIM expression in response to ER stress. PLoS One.

[23] Galehdar Z, Swan P, Fuerth B, Callaghan SM, Park DS, Cregan SP (2010). Neuronal apoptosis induced by endoplasmic reticulum stress is regulated by ATF4-CHOP-mediated induction of the Bcl-2 homology 3-only member PUMA. J Neurosci.

[24] Oyadomari S, Mori M (2004). Roles of CHOP/GADD153 in endoplasmic reticulum stress. Cell Death Differ.

[25] Slemmer Jennifer, Weber John (2014). Assessing Antioxidant Capacity in Brain Tissue: Methodologies and Limitations in Neuroprotective Strategies. Antioxidants.

[26] Behl C, Moosmann B (2002). Antioxidant neuroprotection in Alzheimer's disease as preventive and therapeutic approach. Free Radic Biol Med.

[27] Essa MM, Vijayan RK, Castellano-Gonzalez G, Memon MA, Braidy N, Guillemin GJ (2012). Neuroprotective effect of natural products against Alzheimer's disease. Neurochem Res.

[28] Leong PK, Chiu PY, Chen N, Leung H, Ko KM (2011). Schisandrin B elicits a glutathione antioxidant response and protects against apoptosis via the redox-sensitive ERK/Nrf2 pathway in AML12 hepatocytes. Free Radic Res.

[29] Sun Z, Huang Z, Zhang DD (2009). Phosphorylation of Nrf2 at multiple sites by MAP kinases has a limited contribution in modulating the Nrf2-dependent antioxidant response. PLoS One.

[30] Chang L, Karin M (2001). Mammalian MAP kinase signalling cascades. Nature.

[31] Li J (2013). O W, Li W, Jiang ZG, Ghanbari HA: **oxidative stress and neurodegenerative disorders**. Int J Mol Sci.

[32] Stanciu M, DeFranco DB (2002). Prolonged nuclear retention of activated extracellular signal-regulated protein kinase promotes cell death generated by oxidative toxicity or proteasome inhibition in a neuronal cell line. J Biol Chem.

[33] Di Giacomo C, Acquaviva R, Santangelo R, Sorrenti V, Vanella L, Li Volti G, D'Orazio N, Vanella A, Galvano F (2012). Effect of treatment with Cyanidin-3-O-β-D-Glucoside on rat ischemic/reperfusion brain damage. Evid Based Complement Alternat Med : eCAM.

[34] Fang J (2014). Bioavailability of anthocyanins. Drug Metab Rev.

[35] Marczylo Timothy H., Cooke Darren, Brown Karen, Steward William P., Gescher Andreas J. (2009). Pharmacokinetics and metabolism of the putative cancer chemopreventive agent cyanidin-3-glucoside in mice. Cancer Chemotherapy and Pharmacology.

[36] Shih Ping-Hsiao, Yeh Chi-Tai, Yen Gow-Chin (2005). Effects of anthocyanidin on the inhibition of proliferation and induction of apoptosis in human gastric adenocarcinoma cells. Food and Chemical Toxicology.

[37] Xu M, Bower KA, Wang S, Frank JA, Chen G, Ding M, Wang S, Shi X, Ke Z, Luo J (2010). Cyanidin-3-Glucoside inhibits ethanol-induced invasion of breast cancer cells overexpressing ErbB2. Mol Cancer.

[38] Andres-Lacueva C, Shukitt-Hale B, Galli RL, Jauregui O, Lamuela-Raventos RM, Joseph JA (2005). Anthocyanins in aged blueberry-fed rats are found centrally and may enhance memory. Nutr Neurosci.

[39] Mazza G, Kay CD, Cottrell T, Holub BJ (2002). Absorption of anthocyanins from blueberries and serum antioxidant status in human subjects. J Agric Food Chem.

[40] Milbury PE, Kalt W (2010). Xenobiotic metabolism and berry flavonoid transport across the blood-brain barrier. J Agric Food Chem.

[41] Chen Gang, Bower Kimberly A., Xu Mei, Ding Min, Shi Xianglin, Ke Zun-Ji, Luo Jia (2009). Cyanidin-3-Glucoside Reverses Ethanol-Induced Inhibition of Neurite Outgrowth: Role of Glycogen Synthase Kinase 3 Beta. Neurotoxicity Research.

[42] Chen G, Ma C, Bower KA, Shi X, Ke Z, Luo J (2008). Ethanol promotes endoplasmic reticulum stress-induced neuronal death: involvement of oxidative stress. J Neurosci Res.

[43] Zhu W, Jia Q, Wang Y, Zhang Y, Xia M (2012). The anthocyanin cyanidin-3-O-beta-glucoside, a flavonoid, increases hepatic glutathione synthesis and protects hepatocytes against reactive oxygen species during hyperglycemia: involvement of a cAMP-PKA-dependent signaling pathway. Free Radic Biol Med.

[44] Fratantonio D, Speciale A, Ferrari D, Cristani M, Saija A, Cimino F (2015). Palmitate-induced endothelial dysfunction is attenuated by cyanidin-3-O-glucoside through modulation of Nrf2/Bach1 and NF-kappaB pathways. Toxicol Lett.

[45] Fukumoto LR, Mazza G (2000). Assessing antioxidant and prooxidant activities of phenolic compounds. J Agric Food Chem.

[46] Panee J, Liu W, Nakamura K, Berry MJ (2007). The responses of HT22 cells to the blockade of mitochondrial complexes and potential protective effect of selenium supplementation. Int J Biol Sci.

[47] Cullinan SB, Diehl JA (2006). Coordination of ER and oxidative stress signaling: the PERK/Nrf2 signaling pathway. Int J Biochem Cell Biol.

[48] Fricker M, Tolkovsky AM, Borutaite V, Coleman M, Brown GC (2018). Neuronal cell death. Physiol Rev.

[49] Chhunchha B, Fatma N, Kubo E, Rai P, Singh SP, Singh DP (2013). Curcumin abates hypoxia-induced oxidative stress based-ER stress-mediated cell death in mouse hippocampal cells (HT22) by controlling Prdx6 and NF-kappaB regulation. Am J Physiol Cell Physiol.

[50] Zhang Q, Liu J, Chen S, Liu J, Liu L, Liu G, Wang F, Jiang W, Zhang C, Wang S (2016). Caspase-12 is involved in stretch-induced apoptosis mediated endoplasmic reticulum stress. Apoptosis : an international journal on programmed cell death.

[51] Valko M, Leibfritz D, Moncol J, Cronin MT, Mazur M, Telser J (2007). Free radicals and antioxidants in normal physiological functions and human disease. Int J Biochem Cell Biol.

[52] Prior RL, Wu X (2006). Anthocyanins: structural characteristics that result in unique metabolic patterns and biological activities. Free Radic Res.

[53] Tan L, Yang HP, Pang W, Lu H, Hu YD, Li J, Lu SJ, Zhang WQ, Jiang YG (2014). Cyanidin-3-O-galactoside and blueberry extracts supplementation improves spatial memory and regulates hippocampal ERK expression in senescence-accelerated mice. Biomedical and environmental sciences : BES.

[54] Faria A, Pestana D, Teixeira D, Azevedo J, De Freitas V, Mateus N, Calhau C (2010). Flavonoid transport across RBE4 cells: a blood-brain barrier model. Cellular & molecular biology letters.

[55] Fornasaro S, Ziberna L, Gasperotti M, Tramer F, Vrhovšek U, Mattivi F, Passamonti S (2016). Determination of cyanidin 3-glucoside in rat brain, liver and kidneys by UPLC/MS-MS and its application to a short-term pharmacokinetic study. Sci Rep.

[56] Kalt W, Blumberg JB, McDonald JE, Vinqvist-Tymchuk MR, Fillmore SA, Graf BA, O'Leary JM, Milbury PE (2008). Identification of anthocyanins in the liver, eye, and brain of blueberry-fed pigs. J Agric Food Chem.

[57] Talavera S, Felgines C, Texier O, Besson C, Gil-Izquierdo A, Lamaison JL, Remesy C (2005). Anthocyanin metabolism in rats and their distribution to digestive area, kidney, and brain. J Agric Food Chem.

[58] Kraft AD, Johnson DA, Johnson JA (2004). Nuclear factor E2-related factor 2-dependent antioxidant response element activation by tert-butylhydroquinone and sulforaphane occurring preferentially in astrocytes conditions neurons against oxidative insult. J Neurosci.

[59] Shih AY, Johnson DA, Wong G, Kraft AD, Jiang L, Erb H, Johnson JA, Murphy TH (2003). Coordinate regulation of glutathione biosynthesis and release by Nrf2-expressing glia potently protects neurons from oxidative stress. J Neurosci.

[60] Wang Q, Chuikov S, Taitano S, Wu Q, Rastogi A, Tuck SJ, Corey JM, Lundy SK, Mao-Draayer Y (2015). Dimethyl Fumarate protects neural stem/progenitor cells and neurons from oxidative damage through Nrf2-ERK1/2 MAPK pathway. Int J Mol Sci.

